RETRACTED

# Dioscin induces prostate cancer cell apoptosis through activation of estrogen receptor-*β*

**DOI:** 10.1038/cddis.2017.391

**Published:** 2017-08-10

**Authors:** Xufeng Tao, Lina Xu, Lianhong Yin, Xu Han, Yan Qi, Youwei Xu, Shasha Song, Yanyan Zhao, Jinyong Peng

**Affiliations:** 1 College of Pharmacy, Dalian Medical University, Western 9 Lvshunnan Road, Dalian 116044, China

## Abstract

Recent researches have shown that estrogen receptor-*β* (ER*β*) activator may be a potent anticancer agent for prostate cancer (PCa), and our previous study also indicated that dioscin can upregulate the expression of ER*β* in MC3T3-E1 cell. In the present work, the activity and mechanism of dioscin, a natural product, against PCa were investigated. The results showed that dioscin markedly inhibited cell viability, colony formation, motility and induced apoptosis in PC3 cells. Moreover, dioscin disrupted the formation of PC3 cell-derived mammospheres and reduced aldehyde dehydrogenase (ALDH) level and the CD133^+^/CD44^+^ cells, indicating that dioscin had a potent inhibitory activity on prostate cancer stem cells (PCSCs). *In vivo* results also showed that dioscin significantly suppressed the tumor growth of PC3 cell xenografts in nude mice. Furthermore, mechanism investigation showed that dioscin markedly upregulated ER*β* expression level, subsequently increased prolyl hydroxylase 2 level, decreased the levels of hypoxia-inducible factor-1*α*, vascular endothelial growth factor A and BMI-1, and thus induced cell apoptosis by regulating the expression levels of caspase-3 and Bcl-2 family proteins. In addition, transfection experiment of ER*β*-siRNA further indicated that diosicn showed excellent activity against PCa *in vitro* and *in vivo* by increasing ER*β* expression level. The co-immunoprecipitation (Co-IP) results further suggested that dioscin promoted the interaction of c-ABL and ER*β*, but did not change c-ABL expression. Moreover, the molecular docking assay showed that dioscin processed powerful affinity toward to ER*β* mainly through the strong hydrogen bonding and hydrophobic effects, and the actions of dioscin on ER*β* activation and tumor cells inhibition were significantly weakened in the mutational (Phe-336, Phe-468) PC3 cells. Collectively, these findings proved that dioscin exerted efficient anti-PCa activity via activation of ER*β*, which should be developed as an efficient candidate in clinical for treating this cancer in the future.

Prostate cancer (PCa), the second most common cause of cancer death, is the most commonly diagnosed malignancy in males.^1^ Only in the year of 2015, over 365 000 patients succumbed to death by PCa all over the world.^2^ In China, PCa ranked the ninth with an incidence of 7.10/10^5^ populations among all cancers according to the National Central Cancer Registry of China 2015 Annual Report.^3^ Androgens are pivotal both for the development and function of normal prostate and for the maintenance of cancer cells that come from the secretory epithelium of prostate.^4^ Therefore, PCa initially depends on androgen deprivation therapy and bilateral orchiectomy leads to a temporary inhibition of tumor growth, but the cancer finally develops resistance to these therapies and will progress to castration-resistant PCa with the growth ability.^5^ Despite the high morbidity and mortality of PCa, the majority of patients are initially treated with radiation or surgery.^5^ Moreover, there is no effective therapy for PCa once it has spread beyond the prostate.^6^ Therefore, more works should be devoted for reducing the occurrence and impact of this disease.

RETRACTED

Estrogen receptor is very important for prostate development, which includes two forms: estrogen receptor-*α* (ER*α*) and estrogen receptor-*β* (ER*β*). ER*α* exists in stroma, and it occurs in ductal epithelial cells when the duct branches. However, it is seldom present in the adult prostate, in which ER*β* is the most abundant ER subtype.^7, 8^ ER*β* is massively expressed in the secretory cavity and basement of benign prostate epithelium as well as in the infiltrating immune cells and the stroma.^9^ The proposed functions of ER*β* include anti-proliferative effect, pro-differentiative action, regulating apoptosis and controlling antioxidant gene expression.^10^ Moreover, ER*β* expression decreases in localized PCa with increasing grade through low to high Gleason scores, which indicates that ER*β* maybe a tumor suppressor gene.^11^ The mechanism involves the ability of ER*β* to maintain prolyl hydroxylase 2 (PHD2) protein expression and subsequently advance hypoxia-inducible factor (HIF)-1*α* degradation.^12^ Previous researches have indicated that loss of HIF-1*α* can inhibit autocrine vascular endothelial growth factor A (VEGF-A) signaling, which is emerged as a key component that involves in the apoptosis and motility of tumor cells.^13, 14^ Therefore, the activation of ER*β* signal maybe a potent therapeutic method for PCa by inducing tumor cell apoptosis and reducing its motility. Of particular relevance, the suppressed VEGF-A signaling conversely results in the upregulation of ER*β* by inhibiting the expression of BMI-1 polycomb ring finger oncogene (BMI-1), which is a transcriptional repressor of ER*β*.^15, 16, 17^

Traditional Chinese medicines (TCMs) with the abundant sources of biologically active substances have been widely used to protect health and control diseases in clinical practices.^18^ Some natural products including ailanthone, cucurbitacin B and flavonolignans from medicinal plants have potent effects against PCa.^19, 20, 21^ Therefore, it is reasonable to explore effective natural products from TCMs to treat PCa.

RETRACTED

Dioscin (the chemical structure is shown in Supplementary Figure S1) is a typical multi-effect natural product that exists in some medicinal herbs,^22^ and some TCMs including Liuwei Dihuang decoction (LW) and Di’ao Xinxuekang (Di’ao XXK), which have been clinically used to treat various diseases.^23, 24^ Pharmacological studies have shown that dioscin processes anti-cerebral ischemia/reperfusion injury,^25^ anti-liver fibrosis,^26, 27, 28^ anti-obesity^29^ and anticancer effects.^30, 31, 32, 33^ Moreover, our previous researches have shown that dioscin can upregulate the level of ER*β* in preosteoblast MC3T3-E1 cells.^34^ Importantly, previous work also proved that dioscin had potential anti-tumor activity in androgen-dependent human PCa cell line-LNCaP cell by activating apoptosis pathway, which might be associated with caspase-3 and Bcl-2 protein family.^35^ However, the deeply mechanisms and anti-pancreatic cancer activity on androgen-independent human PCa cell line-PC3 cells have not been reported. Moreover, the effects of dioscin on prostate cancer stem cells (PCSCs) and its drug-target also remain unknown in our best knowledge.

Therefore, the aim of this paper was to investigate the effects of dioscin against PCa, and then the mechanism associated with ER*β* signal pathway was also studied. The findings may provide novel insights and develop a potent candidate for preventing and treating PCa.

## Results

### Effects of dioscin on cytotoxicity of PC3 cells and mammospheres formation

Cell viabilities results showed that the half maximal inhibitory concentrations (IC_50_) of dioscin at 24 h were 5.6 *μ*M and 10.0 *μ*M in PC3 cells and PC3-derived mammosphere, respectively (Figure 1a), which suggested that dioscin could markedly suppress both PC3 monolayer and mammosphere growth. In addition, the cell morphologies were observed by a light microscope and the results revealed that dioscin obviously caused PC3 cell death (Figure 1b), and disrupted the PC3-derived mammospheres formation (Figure 1c). Aldehyde dehydrogenase (ALDH) is a fine cancer stem cell marker which can be assayed by Aldefluor staining kit. Using fluorescence microscopy, we identified ALDH-positive cells with green color, and dioscin at the dose of 10.0 *μ*M obviously inhibited mammospheres formation (Figure 1d).

### Dioscin inhibited colony formation and motility in PC3 cells, and reduced CD133^+^/CD44^+^ cells in mammospheres

The proliferation, migration and invasion capacities of cells are the three most critical characteristics of malignant cell behavior.^36^ As shown in Figure 2a, the action of dioscin on PC3 cells proliferation was also determined through colony formation assay, and the results showed that dioscin (1.4, 2.8 and 5.6 *μ*M) caused significant decrease in colony formation in PC3 cells. In addition, the results of cell scratch test indicated that dioscin at the low concentrations (0.35, 0.7 and 1.4 *μ*M) showed slower rates of wound healing, and reduced cell migration of PC3 cells compared with control group (Figure 2b). More importantly, PCSCs can preferentially express cell surface and transmembrane proteins, including CD44 and CD133. In the present work, the results of flow-cytometric assay showed that the percentage of the cells stained for CD133^+^/CD44^+^ in mammospheres was potently increased compared with PC3 monolayer, which was significantly decreased by dioscin at the dose of 10.0 *μ*M (Figure 2c). These data suggested that dioscin had the capacity to inhibit the growth of PC3 cells and PCSCs.

RETRACTED

### Dioscin-induced apoptosis in PC3 cells

To further explore the mechanism of dioscin-induced the inhibition of cell proliferative, the results of flow cytometry assay demonstrated that dioscin markedly increased the relative amount of cell apoptosis. As shown in Figure 3a, the apoptotic rates were significantly increased from 8.11% (control group) to 12.67%, 14.25% and 17.86% in PC3 cells treated with dioscin (1.4, 2.8 and 5.6 *μ*M) for 24 h, respectively. Moreover, in PC3-derived mammospheres, the apoptotic rates were notably increased from 7.62% (control group) to 10.62%, 11.58% and 15.67% treated by dioscin (2.5, 5.0 and 10.0 *μ*M) for 24 h, respectively (Figure 3b). In addition, compared with control cells, dioscin significantly induced caspase substrate (polyADP-ribose polymerase (PARP) and caspase-3) cleavage, upregulated Bcl-2-associated X protein (Bax) and downregulated B-cell CLL/lymphoma 2 (Bcl-2) expression levels in PC3 cells (Figure 3c) and PC3-derived mammospheres (Figure 3d) with a dose-dependent manner (the statistical analysis is shown in Supplementary Figures S2a-b).

### Dioscin activated ER*β* signaling pathway in PC3 cells and mammospheres

To determine the effect of dioscin on ER*β* signaling, PC3 cells and mammospheres were treated with different concentrations of disocin. We found that the protein levels of ER*β*, PHD2 were significantly upregulated, and the protein levels of HIF-1*α* and VEGF-A were markedly downregulated by dioscin compared with control groups both in PC3 cells (Figure 4a) and PC3-derived mammospheres (Figure 4b). These data suggested that dioscin inhibited VEGF-A signaling pathway by activating ER*β*. Furthermore, as shown in Figures 4c and d and Supplementary Figures S3a-b, compared with control cells, dioscin notably decreased BMI-1 protein expression in PC3 cells and mammospheres.

RETRACTED

### ER*β*-siRNA abrogated the inhibitory effects of dioscin on PC3 cells

To explore the role of ER*β* in anticancer activity of dioscin, the ER*β*-siRNA transfection approach *in vitro* was tested. As shown in Figure 5a, ER*β*-siRNA markedly promoted PC3 monolayer growth, which was notably inhibited by dioscin at the dose of 5.6 *μ*M. Moreover, pretreatment of ER*β*-siRNA plus dioscin also increased PC3 monolayer growth with no significant difference compare with ER*β*-siRNA group, which indicated that ER*β*-siRNA abrogated the inhibitory effect of dioscin on PC3 cells. Similarly, the effects of dioscin (5.6 *μ*M) on colony formation, motility and apoptosis in PC3 cells were all abrogated by ER*β*-siRNA (Figures 5b and d). In addition, after transfecting with ER*β*-siRNA at the presence or absence of dioscin, the expression levels of cleaved caspase-3, cleaved PARP and Bax were all notably decreased and the Bcl-2 expression level was markedly increased compared with control group (Figure 6a). As the same, compared with control group, the protein levels of ER*β* and PHD2 were notably downregulated, and the levels of HIF-1*α*, VEGF-A and BMI-1 were markedly upregulated after transfecting with ER*β*-siRNA at the presence or absence of dioscin (Figure 6b and Supplementary Figure S4a). These results suggested that ER*β*-siRNA transfection abrogated the activation effect of dioscin on ER*β* signaling pathway.

### Dioscin inhibited tumor growth of cell xenografts in nude mice

We used a PC3 cell tumor xenograft model to evaluate the *in vivo* anticancer and ER*β* activation of dioscin, and the data showed that dioscin significantly inhibited tumor growth in mice (Figure 7a). As shown in Figure 7b, the results indicated that dioscin at the dose of 80 mg/kg notably decreased tumor volumes by 68.2% and tumor weight by 67.1% in nude mice transplanted with PC3 cells. However, ER*β*-siRNA transfection increased the tumor volumes and weight with or without dioscin, suggesting that ER*β*-siRNA abrogated the inhibitory effects of dioscin on tumor growth *in vivo*. In addition, more cell injury and fewer cells were observed in dioscin-treated group compared with control group basing on hematoxylin–eosin (HE) staining, and ER*β*-siRNA transfection abrogated the action of dioscin on HE staining (Figure 7c).

### Dioscin increased ER*β* expression and induced apoptosis *in vivo*

To test the effect of ER*β* activation and cell apoptosis on the anticancer activity of dioscin *in vivo*, we measured the changes of ER*β* expression and cell apoptosis in response to ER*β*-siRNA through immunofluorescence and terminal deoxynucleotidyl transferase dUTP nick-end labeling (TUNEL) assay. As shown in Figure 7d, compared with control group, ER*β* protein expression and TUNEL-positive cells were all obviously increased in the tumor tissue of dioscin-treated mice. At the presence or absence of dioscin after transfecting with ER*β*-siRNA, ER*β* protein expression and TUNEL-positive cells were notably decreased. Therefore, dioscin-induced cell apoptosis *in vivo* mainly by increasing ER*β* expression level.

RETRACTED

### Effects of dioscin on ER*β* signaling were abrogated by ER*β*-siRNA *in vivo*

To validate the modulation of tumor apoptosis by dioscin via ER*β* signaling, we treated the mice with ER*β*-siRNA in the presence or absence of dioscin. The results indicated that dioscin-induced cell apoptosis mainly by adjusting caspase-3/PARP and Bax/Bcl-2 signals (Figure 8a). Moreover, ER*β*-siRNA abolished the effects of dioscin on ER*β* pathway *in vivo* via affecting the expression levels of ER*β*, PHD2, HIF-1*α*, VEGF-A and BMI-1 (Figure 8b and Supplementary Figure S4b).

### Dioscin promoted the interaction of c-ABL and ER*β*

BCR Abelson tyrosine kinase (c-ABL) can enhance the anti-tumor action of ER*β* by directly controlling the status of phosphotyrosine residue (Y36). To further elucidate the effects of dioscin on ER*β*, we carried out the Co-IP assay. As shown in Figure 9a, the results of ‘Input experiment’ showed that dioscin (5.6 *μ*M) had no obvious effect on c-ABL protein expression in PC3 cells. However, the ‘Co-IP experiment’ showed that c-ABL antibody could pull down the protein level of ER*β* instead of ER*α*, and dioscin significantly enhanced this action. These results indicated that dioscin promoted the interaction of c-ABL and ER*β*, but did not change c-ABL expression.

### Dioscin directly targeted with ER*β*

In order to predict the drug-target of dioscin against prostatic cancer, molecular docking assay was used. The three-dimensional structure of dioscin and the crystal structure of ER*β* (PDB, ID: 2YLY) are shown in Supplementary Figures S5a-b, and the active pocket of ER*β* protein is shown in Supplementary Figure S5c. The binding mode of dioscin and ER*β* is shown in Figure 9b. The results indicated that the root-mean-square deviation and binding energy of the optimal docking conformation of dioscin and ER*β* were 1.13 Å and −7.98 kcal/mol, respectively. Moreover, the hydrogen bond model of dioscin and ER*β* are shown in Figure 9b, and the analyses of hydrogen bonding and hydrophobic effects indicated that the amino-acid residues involved in the formation of hydrogen bonds included methionine-336 (Met-336) and alanine-468 (Ala-468). The hydrophobic bond formation between the condensed ring long chain of dioscin- molecule and the hydrophobic residues within ER*β* active pocket involved Leucine- 301 (Leu-301), alanine-302 (Ala-302), glutamic acid-305 (Glu-305), leucine-339 (Leu-339) and arginine-346 (Arg-346), which further enhanced the combination of dioscin and ER*β*. These results indicated that dioscin processed powerful affinity toward to ER*β* mainly through the strong hydrogen bonding and hydrophobic effects.

RETRACTED

### Mutation assay

To validate the modulation of tumor cell by dioscin via the activation of ER*β*, we detected the ER*β* protein expression and cell viability in PC3 cells after transfecting the mutational-ER*β* cDNA (Phe-336, Phe-468). As shown in Figure 9c, the up- regulation of dioscin on ER*β* was significantly decreased in the mutant type (MT) cells. Moreover, the assay of cell viability showed that dioscin could also induce cell death in MT-PC3 cells. However, the inhibition of dioscin was also markedly decreased compared with the wild-type (WT)-PC3 cells (Figure 9d).

## Discussion

PCa is a malignant tumor with high morbidity and high mortality, and there is lack of effective therapies.^5^ Dioscin is a natural product that processes beneficial actions against colon cancer,^30^ glioblastoma multiforme,^31^ pancreatic cancer^32^ and lung cancer^33^ in our previous studies. Therefore, we explored whether dioscin has potent effect against PCa on androgen-independent human PCa cell line-PC3 in this study. The results in this paper showed that dioscin notably suppressed cell viability and colony formation with IC_50_ value at 5.6 *μ*M. Moreover, to observe the effects of dioscin on cell migration and invasion, we used dioscin at the concentrations of 0.35, 0.7 and 1.4 *μ*M, the results showed that dioscin reduced cell migration and invasion in PC3 cells. Previous work has shown that one efficient anticancer therapy is to increase the percentage of tumor cells undergoing apoptosis, which is a ‘suicide’ program for the cells to cause minimal injury to surrounding tissues.^37^ Therefore, we detected the action of dioscin on PC3 cells apoptosis using flow cytometry assay, and found that dioscin had the ability to induce the apoptosis in PC3 cells.

In addition, PCSCs are the cell origin of PCa and have an important role in the progression to PCa.^38^ PCSCs constitute a very small proportion of tumor cell population, which are characterized by high levels of ALDH activity.^39^ Moreover, ALDH is a fine cancer stem cell marker which can be assayed by Aldefluor staining kit. In this paper, the Aldefluor/Hoechst 33342 double-staining results indicated that dioscin at the concentration of 10.0 *μ*M disrupted the mammospheres formation and decreased PCSCs. Moreover, PCSCs can preferentially express cell surface and transmembrane proteins including CD44 and CD133 in PCa,^40^ and the present results showed that dioscin markedly decreased CD133^+^/CD44^+^ cells and induced cell apoptosis in PC3 mammospheres. Therefore, dioscin showed the potent inhibitory activity on PCSCs. Meanwhile, *in vivo* experiments also indicated that dioscin at the dose of 80 mg/kg notably decreased tumor volumes by 68.2% and tumor weight by 67.1% in nude mice transplanted with PC3 cells after 21 days of treatment. In general, the above results indicated that dioscin showed active effects against PCa *in vitro* and *in vivo*.

RETRACTED

Some reports have demonstrated that repression of ER*β* is an integral component for the prostate tumorigenesis.^41^ In detail, loss of ER*β* stabilizes HIF-1*α* and enables autocrine VEGF-A signaling by reducing the enzymatic activity of PHD2, which is the pivotal hydroxylation enzyme of HIF-1*α*.^11^ As we know, HIF-1*α*/VEGF-A signaling is emerged as a crucial component that involves in the motility and inducing of apoptosis in tumor cells.^15^ Therefore, activation of ER*β* can promote cell apoptosis and reduce cell migration and invasion contributing to its anticancer potential. In the present work, our results indicated that dioscin significantly increased the expression levels of ER*β* and PHD2, decreased the levels of HIF-1*α* and VEGF-A, and induced apoptosis via adjusting caspases-3 and Bax/Bcl-2 signals *in vitro* and *in vivo*. In addition, BMI-1 is an important oncogenic factor in PCa as the transcriptional repressor of ER*β*, which can be triggered by HIF-1*α*/VEGF-A signals.^16^ In this study, the results showed that dioscin markedly inhibited the protein expression of BMI-1. Finally, as shown in Supplementary Figure S6, the anti-PCa effect of dioscin may result primarily from ER*β* activation.

To further validate the action of dioscin against PCa through ER*β* pathway, the ER*β*-siRNA *in vitro* and *in vivo* were used. The results indicated that ER*β*-siRNA abrogated the effects of dioscin on PC3 monolayer growth, colony formation, apoptosis and migration. In addition, the *in vivo* experiments further showed that ER*β*-siRNA transfection increased the tumor volume and weight at the presence or absence of dioscin, which indicated that ER*β*-siRNA abrogated the inhibitory effects of dioscin on tumor growth *in vivo*. The similar results were obviously observed in the expression levels of cleaved caspases-3 and PARP, and ER*β* signaling related proteins including ER*β*, PHD2, HIF-1*α*, VEGF-A and BMI-1 *in vitro* and *in vivo*. Therefore, the above data further suggested the anti-PCa activity of dioscin involved in ER*β* activation.

c-ABL protein is a transcription coregulator with efficient tyrosine phosphatase activity. Latest research has shown that c-ABL can enhance the anti-tumor action of ER*β* by directly controlling the status of phosphotyrosine residue (Y36).^17^ Therefore, regulation of c-ABL/ER*β* signal maybe one potent therapeutic method for PCa. Based on our investigation, the Co-IP results indicated that dioscin promoted the interaction of c-ABL and ER*β*, but did not change c-ABL expression. Moreover, the molecular docking assay further showed that dioscin processed powerful affinity toward to ER*β* mainly through the strong hydrogen bonding and hydrophobic effects. In order to further confirm the effects of hydrogen bonding on activation of ER*β* by dioscin, the results of amino-acid mutation experiments showed that the activation of ER*β* and the inhibition of cell viability by dioscin were significantly decreased after transfecting with mutational-ER*β* cDNA (Phe-336, Phe-468) in PC3 cells.

RETRACTED

Therefore, these findings in this paper provided novel insight into the molecular mechanism of dioscin against PCa and suggested that dioscin should be developed as an efficient candidate in clinical for treating this cancer in the future. Dioscin is also one major active ingredient in LW and Di’ao XXK, which have been widely used to treat various diseases clinically.^23, 24^ Therefore, our results may expand the clinical applications of the related-Chinese patent medicines to prevent and treat PCa. Of course, further researches are required to thoroughly elucidate the activities, mechanisms and clinical applications of this compound against PCa.

## Materials and methods

### Chemicals and materials

Dioscin was purchased from Shanghai Tauto Biotech Co., Ltd, (Shanghai, China), which was added into the medium through dissolving with DMSO with final concentration of <0.1% in cell experiments, or suspended in 0.5% sodium carboxyl methyl cellulose (CMC-Na) in animal experiments. Protein Extraction kit, penicillin and streptomycin combination were purchased from KeyGEN BioTECH (Naijing, China). Bicinchoninic acid (BCA) protein assay kit was obtained from Beyotime Institute of Biotechnology (Jiangsu, China). CMC-Na, Tris (hydroxymethyl) aminomethane (Tris) and sodium dodecyl sulfate (SDS) were purchased from Sigma (Santa clara, CA, USA). ER-siRNA that used *in vitro* and chemically modified ER*β*- siRNA used *in vivo* were all purchased from RiboBio Co., Ltd. (Guangzhou, China).

RETRACTED

### Cell lines and cell culture

The PC3 cell line was purchased from Zhong Qiao Xin Zhou Biotechnology Co., Ltd. (Shanghai, China) and cultured in Dulbecco's minimum essential medium (DMEM)/F12 medium (Hyclone, Logan, UT, USA) supplemented with 10% fetal bovine serum (FBS) (Hyclone) and 1% penicillin and streptomycin combination. The cells grew in standard cell culture conditions (5% CO_2_, 95% humidity) at 37 °C.

### *In vitro* culture of mammospheres

The PC3 cells were used to generate mammospheres using the complete MammoCult Human Medium (MammoCult basal Medium: MammoCult proliferation supplement=9:1) (STEMCELL Technologies, Vancouver, BC, Canada). To culture the second generation mammospheres, the first generation mammospheres were harvested by trypsinization and mechanically dispersed by gentle pipetting. Single-cell suspensions were observed microscopically, and the cells were counted and re-suspended in fresh MammoCult medium. Mammospheres were exposed to given different treatments after 5 days of culturing.

### Determination of cell viabilities and morphological changes

The PC3 cells were seeded in 96-well plates (5000 cells/well) in DMEM/F12 medium and incubated overnight, and the PC3 cell-derived mammospheres were seeded in growth medium for 5 days culturing. Subsequently, various concentrations of dioscin (0.18–92 *μ*M for PC3 monolayers; 0.36–184 *μ*M for mammospheres) were added in each well. After PC3 cells were incubated for 24 h, the cell viability was analyzed using the MTT assay kit (Beyotime, Jiangsu). Alternatively, cytotoxicity of dioscin on PC3 cell-derived mammospheres was evaluated using the CCK-8 assay kit (Beyotime). Similarly, in order to observe the morphologies of PC3 and mammospheres, various concentrations of dioscin (1.4, 2.8 and 5.6 *μ*M for PC3 cells; 2.5, 5.0 and 10.0 *μ*M for mammospheres) was added in the cells medium for 24 h culturing. The morphologies were visualized using an inverted microscope (Nikon, Chiyoda pill, Tokyo, Japan).

### ALDH assay

The second generation mammospheres were treated with dioscin (10 *μ*g/ml) for 24 h. Then, the cells were collected and re-suspended in 0.5 ml PBS. At last, the cells were incubated using 5 *μ*g/ml of Aldefluor staining solution (STEMCELL Technologies) for 1 h at 37 °C and then counterstained with 10 *μ*g/ml of Hoechst 33342 (Solarbio, Beijing, China) for 10 min. Images were captured using a laser scanning confocal microscope (Leica, Wetzlar, Hesse, Germany) with × 800 magnification.

RETRACTED

### Colony formation assay

The PC3 cells were harvested, and single cells were seeded (500 cells/well) into six-well plates, and then treated with different concentrations of dioscin (1.4, 2.8 and 5.6 *μ*M) once every 3 days and grown for 6 days. Finally, the colonies were stained with hematoxylin solution for 10 min at room temperature, and the images were photographed by a digital camera.

### Scratch assay

Cell migration and invasion abilities were detected using scratch assay. In order to minimize the impact of the differential cell growth rates on the motility determination, we induced cell cycle arrest by keeping cells under serum starvation conditions for 24 h before implementing the scratch assay. The cells were grown to 80% confluency in six-well plates and then were wounded with a sterile 100 *μ*l pipette tip on the cell monolayers and washed with serum-free medium to remove detached cells. Next, the cells were treated with low concentrations of dioscin (0.35, 0.7 and 1.4 *μ*M) for 24 h continuous cultivation. Finally, the images of wound gap were photographed using an inverted microscope.

### Transwell migration assay

Cell migration and invasion were also measured using sterile Transwell with 8.0 *μ*m pore polycarbonate membrane insert (Corning Incorporated, Corning, NY, USA). Similarly, after maintaining PC3 cells under serum starvation conditions for 24 h, the cells (2 × 10^4^ cells/well) were digested and loaded onto the top of a 24-well migration chamber in 100 *μ*l serum-free DMEM/F12 medium containing different low concentrations of dioscin (0.35, 0.7 and 1.4 *μ*M), and 0.75 ml medium containing 10% FBS was added to the lower chamber for 24 h culturing. Eventually, the cells that had migrated into the lower surface of the filter were fixed with 10% formaldehyde and stained with hematoxylin after 24 h incubation.

### Determination of CD133^+^/CD44^+^ cells

Flow cytometry was used to identify of the markers of PCSCs. In detail, PC3 cells, PC3-derived mammospheres and dioscin-treated PC3-derived mammospheres were harvested and re-suspended in 500 *μ*l of PBS. Next, 10 *μ*l of anti-CD133/1-PE and 10 *μ*l of anti-CD44-FITC monoclonal antibodies (Miltenyi Biotec Technology & Trading, Teterow, Germany) were added. The mixture was incubated at room temperature for 20 min in the darkroom. Finally, the FACS Calibur (Becton-Dickinson, Franklin Lake, NJ, USA) was used to detect the cells by flow cytometry.

### Apoptosis assay

The PC3 cells and mammospheres were collected and washed three times with ice-cold PBS after treating with different concentrations of dioscin (1.4, 2.8 and 5.6 *μ*M for PC3 cells; 2.5, 5.0 and 10.0 *μ*M for mammospheres) for 24 h. The cells were then stained with 5 *μ*l of Annexin V-FITC and 5 *μ*l of propidium iodide (Beyotime) in 500 *μ*l of binding buffer at room temperature for 10 min in the darkroom according to the manufacturer’s instructions. Eventually, the apoptosis rates of the samples were determined using flow cytometry (Becton-Dickinson).

RETRACTED

### ER*β* siRNA transfection experiments *in vitro*

Transfection was performed to downregulate the ER*β* protein expression level through using ER*β*-siRNA (RiboBio Co. Ltd.), whose sequence is as follows: CAAGGTTTCGAGAGTTAAA. *In vitro* experiment, according to previous methods,^25, 32^ the control-siRNA and ER*β*-siRNA were separately dissolved in Opti-MEM, and then mixed gently with transfection reagent-lipofectamine2000 for 20 min to form siRNA liposomes. The PC3 cells were then transfected with the siRNA liposomes in antibiotic-free cell medium. Finally, cell viabilities, apoptosis, colony formation, motility and the expression levels of ER*β*, PHD2, HIF-1*α*, BMI-1, VEGF-A, cleaved caspase-3 and cleaved polyADP-ribose polymerase (cleaved PARP) were detected after 24 h of transfection in the absence or presence of dioscin (5.6 *μ*M) for an additional 24 h.

### Animal model and experimental protocol

The four-week old BALB/c nude mice (18–22 g) were provided by the Experimental Animal Center at Dalian Medical University (Dalian, China) (SCXK (Liao): 2013-0003). All experiments were approved by the Animal Care and Use Committee of Dalian Medical University, and the procedures were performed in strict accordance with the People’s Republic of China Legislation Regarding the Use and Care of Laboratory Animals. The PC3 cells (4 × 10^5^) were suspended in 100 *μ*l of PBS and injected subcutaneously into the underarm regions of the mice. The animals were then randomly divided into five groups: (1) Control group: the mice were treated with 0.5% CMC-Na; (2) Control-siRNA group: the mice were treated with control-siRNA; (3) Dioscin group: the mice were treated with 80 mg/kg of dioscin; (4) ER*β*-siRNA group: the mice were treated with chemically modified ER-siRNA (200 nmol/kg); (5) ER*β*-siRNA plus dioscin group: the mice were treated with chemically modified ER*β*-siRNA (200 nmol/kg) and dioscin (80 mg/kg); These treatment were begun on day 7 post-inoculation when the tumorigenic rate was 100% in each group and continued for 21 days. Among them, dioscin was suspended in 0.5% CMC-Na and intragastric administrated in mice once a day; chemically modified ER*β*-siRNA was diluted in PBS and intratumoral injected in the mice once every 3 days according to previous methods.^42, 43^ The tumor volumes of mice were measured once every 3 days and calculated using the following formula: *V*=(maximum diameter) × (minimum diameter)^2^/2. The mice were killed after these treatment, the tumors were then peeled and photographed. A part of tumor tissues were fixed in neutral buffered formalin and the others were preserved in the −80°C for following assays.

RETRACTED

### HE staining assay

Formalin-fixed tissues were embedded in paraffin and cut into 5 *μ*m sections. The sections were then stained with HE according to the manufacturer’s instructions, and the images were obtained using a light microscope (Leica) with × 200 magnification.

### ER*β* and TUNEL dual staining assay

The sections were successively pretreated with 0.1% Triton X-100 for 10 min and 5% goat serum albumin for 30 min at 37 °C, and then incubated with anti-ER*β* antibody (1:80, dilution) in a moist box for overnight at 4 °C. The sections were then incubated using a TRITC-conjugated Goat anti-Rabbit IgG (H+L) for 1 h and then incubated with the TUNEL reaction mixture for 1 h at 37 °C according to the manufacturer’s instructions. Finally, the photographs were captured by a fluorescent microscopy (Olympus; Tokyo, Japan) with × 200 magnification.

### Western blotting assay

The total proteins from PC3 cells, PC3 mammospheres and tumor tissues were extracted using cold lysis buffer following standard protocols, and the protein concentrations were detected using a BCA protein assay kit. The protein samples were loaded onto SDS-PAGE gels, separated electrophoretically, and transferred to PVDF membranes (Millipore, Danvers, MA, USA) after they were degenerated using 2 × loading buffer. Then, the membranes were blocked non-specific binding sites with 5% dried skim milk at 37 °C for 1 h, and individually incubated for overnight at 4 °C with primary antibodies (Supplementary Table S1). Finally, the membranes were incubated with horseradish peroxidase-conjugated antibody at room temperature for 2 h. Protein expression levels were then determined using an enhanced chemiluminescence method and imaged by a Bio-Spectrum Gel Imaging System (UVP, Upland, CA, USA). The data were adjusted to correspond internal reference expression (IOD value of target protein *versus* IOD value of GAPDH protein) to eliminate the variations of protein expression.

### Co-IP assay

The PC3 cells and dioscin-treated-PC3 cells grown in regular DMEM/F12 medium were harvested, and the proteins were prepared. One microgram extract was subjected to IP with 2 *μ*g anti-c-ABL antibody as indicated, and the samples were rotated for 4 h at 4 °C. Next, protein G-conjugated sepharose slurry (10 *μ*l) was added in the samples for 2 h rotation. Ultimately, the sepharose beads were washed three times with a high-salt buffer including 20 mM HEPES, 500 mM NaCl, 1% NP-40 and 5 mM EDTA (pH=8.0). Proteins were then analyzed by immunoblotting with either anti-c-ABL or anti-ER*β* polyclonal antibody.

RETRACTED

### Molecular docking assay

The three-dimensional structure of dioscin was drawn by ‘3D Maestro’ software, and then was handled by the ‘prepare_ligand4.py’ script in ‘AutoDock Tools 1.5.6’, which mainly includes the removal of nonpolar hydrogen and giving of the atomic type and gasteiger charge. The crystal structure of ER*β* was extracted by ‘PyMol’ program, and then handled by the ‘prepare_receptor4.py’ script in ‘AutoDockTools 1.5.6’, whose process mainly involved in the removing of crystal water, ions and non-standard amino-acid residues. Next, the docking of ER*β* and dioscin was performed through using of the ‘AutoDock 4.2.6’ program. The binding free energy and the actions of hydrogen bond, hydrophobic, electrostatic were analyzed.

### Mutation assay

Human ER*β* cDNA into pEnter vector was purchased from ViGene BioScieneces, Inc (Rockville, MD, USA), and then mutagenized residues Met-336 and Ala-468 with the Multi Site-Directed Mutagenesis Kit (Qcbio Science & Technologies Co., Ltd, Shanghai, China). We mutated Met-336 to Phe-336 and Ala-468 to Phe-468 in order to decrease intermolecular hydrogen bonding and increase steric hindrance. The according mutant primers (Supplementary Figure S7) were designed using the PrimerX Software (www.bioinformatics.org/primerx/), and synthesized by Invitrogen (Carlsbad, CA, USA). Finally, the effects of dioscin on ER*β* activation and cell death were detected after mutational-ER*β* cDNA was transfect into PC3 cells.

### Statistical analysis

All the data were expressed as mean±S.D. and analyzed using statistical software SPSS 19.0 (IBM, Armonk, NY, USA). Differences among groups were detected through using the one-way analysis of variance, followed by a *post hoc* LSD test, and the comparisons between two groups were performed using an unpaired Student’s *t*-test. *P*<0.05 and *P*<0.01 were considered to be significant.

## Figures and Tables

**Figure 1:** Dioscin exhibited cytotoxicity in PC3 cells, and disrupted mammospheres formation. (**a**) Effects of dioscin on the viabilities of PC3 cells and PC3 cell-derived mammospheres. (**b**) Effects of different concentrations of dioscin (1.4, 2.8 and 5.6 *μ*M) for 24 h on the morphology and structure of PC3 cells (bright-field image). (**c**) Effects of different concentrations of dioscin (2.5, 5.0 and 10.0 *μ*M) for 24 h on the morphology and structure of PC3 cell-derived mammospheres (bright-field image). (**d**) Mammosphere revealing cells staining positive for Aldefluor (green), counterstained with Hoechst 33342 (blue). Data are presented as the mean±S.D. (*n*=6)

**Figure 2:** Dioscin inhibited colony formation and motility in PC3 cells, and reduced the CD133^+^/CD44^+^ cells in mammospheres. (**a**) Effects of dioscin (1.4, 2.8 and 5.6 *μ*M) for 24 h on the colony formation in PC3 cells. (**b**) Effects of dioscin (0.35, 0.7 and 1.4 *μ*M) for 24 h on the cell motility of PC3 cells. (**c**) Effects of dioscin (2.5, 5.0 and 10.0 *μ*M) for 24 h on the CD133^+^/CD44^+^ cells in PC3 cell-derived mammospheres. Data are presented as the mean±S.D. (*n*=5). **P<0.01 *versus* PC3 group; ^##^*P*<0.01 *versus* mammospheres group

**Figure 3:** Dioscin-induced apoptosis in PC3 cells and mammospheres. (**a**) Effects of dioscin (1.4, 2.8 and 5.6 *μ*M) for 24 h on apoptosis of PC3 cells using flow cytometry analysis. (**b**) Effects of dioscin (2.5, 5.0 and 10.0 *μ*M) for 24 h on apoptosis of PC3 cell-derived mammospheres using flow cytometry analysis. (**c**) Effects of dioscin (1.4, 2.8 and 5.6 *μ*M) for 24 h on cleaved caspase-3, cleaved PARP, Bax and Bcl-2 expression levels in PC3 cells. (**d**) Effects of dioscin (2.5, 5.0 and 10.0 *μ*M) for 24 h on cleaved caspase-3, cleaved PARP, Bax and Bcl-2 expression levels in PC3 cell-derived mammospheres. Data are presented as the mean±S.D. (*n*=5).*P<0.05 and **P<0.01 *versus* Control group

**Figure 4:** Dioscin activated ER*β* signaling pathway in PC3 cells and mammospheres. (**a**) Effects of dioscin (1.4, 2.8 and 5.6 *μ*M) for 24 h on ER*β*, PHD2, HIF-1*α* and VEGF-A expression levels in PC3 cells. (**b**) Effects of dioscin (2.5, 5.0 and 10.0 *μ*M) for 24 h on ER*β*, PHD2, HIF-1*α* and VEGF-A expression levels in PC3 cell-derived mammospheres. (**c**) Effect of dioscin (1.4, 2.8 and 5.6 *μ*M) for 24 h on BMI-1 protein expression in PC3 cells. (**d**) Effect of dioscin (2.5, 5.0 and 10.0 *μ*M) for 24 h on BMI-1 protein expression in PC3 cell-derived mammospheres. Data are presented as the mean±S.D. (*n*=5). *P<0.05 and **P<0.01 *versus* Control group

**Figure 5:** Inhibitory effects of dioscin on PC3 cell were abrogated by ER*β*-siRNA. (**a**) Effects of dioscin and ER*β*-siRNA on the viability of PC3 cells. (**b**) Effects of dioscin and ER*β*-siRNA on the colony formation in PC3 cells. (**c**) Effects of dioscin and ER*β*-siRNA on the motility of PC3 cells. (**d**) Effects of dioscin and ER*β*-siRNA on apoptosis in PC3 cells. Data are presented as the mean±S.D. (*n*=6). **P<0.01 *versus* Control group; NS, not significant

**Figure 6:** Effects of dioscin on ER*β* signaling in PC3 cells were abrogated by ER*β*- siRNA *in vitro*. (**a**) Effects of dioscin and ER*β*-siRNA on cleaved caspase-3, cleaved PARP, Bax and Bcl-2 expression levels in PC3 cells. (**b**) Effects of dioscin and ER*β*-siRNA on ER*β*, PHD2, HIF-1*α*, VEGF-A and BMI-1 expression levels in PC3 cells. Data are presented as the mean±S.D. (*n*=5). **P<0.01 *versus* Control group; NS, not significant

**Figure 7:** Dioscin inhibited tumor growth of cell xenografts in nude mice. (**a**) Images of the tumors collected from the mice in different groups. (**b**) Effects of dioscin and ER*β*-siRNA on the mean tumor volumes and weights. (**c**) Effects of dioscin and ER*β*-siRNA on tumor histopathology based on H&E staining (× 200 magnification). (**d**) Effects of dioscin and ER*β*-siRNA on ER*β*/TUNEL double-staining (× 200 magnification). Data are presented as the mean±S.D. (*n*=5). *P<0.05 and **P<0.01 *versus* Control group; NS, not significant

**Figure 8:** Dioscin activated ER*β* signaling *in vivo*. (**a**) Effects of dioscin and ER*β*-siRNA on cleaved caspase-3, cleaved PARP, Bax and Bcl-2 expression levels in tumor tissue. (**b**) Effects of dioscin and ER*β*-siRNA on ER*β*, PHD2, HIF-1*α*, VEGF-A and BMI-1 expression levels in tumor tissue. Data are presented as the mean±S.D. (*n*=5). *P<0.05 and **P<0.01 *versus* Control group; NS, not significant

**Figure 9:** Dioscin promoted the interaction of c-ABL and ER*β*, and directly targeted with ER*β*. (**a**) Effects of dioscin on the interaction of c-ABL and ER*β* in PC3 cells. (**b**) The hydrogen bonding model of dioscin and ER*β*. (**c**) Effect of dioscin on ER*β* expression level in PC3 cells after transfecting with mutational-ER*β* cDNA. (**d**) Effect of dioscin on the cell viability of PC3 cells after transfecting with mutational-ER*β* cDNA. Data are presented as the mean±S.D. (*n*=5). *P<0.05 and **P<0.01 *versus* Vehicle group; ^##^*P*<0.01, Mutant type (MT) *versus* wild-type (WT) group
